The article "Efficacy and Safety of N-Acetylcysteine for Chronic Obstructive Pulmonary Disease and Chronic Bronchitis" was retracted in 2023. Reasons: signs of a paper mill; compromised peer review; unreliable results or conclusions.

# Efficacy and Safety of N-Acetylcysteine for Chronic Obstructive Pulmonary Disease and Chronic Bronchitis

**DOI:** 10.1155/2022/9133777

**Published:** 2022-06-26

**Authors:** Li Zhang, Yan Xiong, Lei Du

**Affiliations:** ^1^Department of Pulmonary Diseases, Wuhan Hospital of Traditional Chinese Medicine, 4300000, China; ^2^Department of Emergency Medicine, Wuhan Hospital of Traditional Chinese Medicine, 4300000, China; ^3^Department of Critical Medicine, Wuhan Hospital of Traditional Chinese Medicine, 4300000, China

## Abstract

**Background:**

Patients with chronic obstructive pulmonary disease (COPD) and chronic bronchitis are associated with poor clinical outcomes. *N*-acetylcysteine (NAC) is a widely used therapeutic option for such patients; however, the clinical efficacy of NAC has not been conclusively determined. We hypothesized that high-dose oral NAC can improve the clinical outcomes for patients with concurrent chronic bronchitis and COPD. *Objective and Methods*. This was a randomized, double-blind, placebo-controlled trial evaluating the efficacy of high-dose NAC for COPD patients with concurrent chronic bronchitis. Study participants were randomized into two groups and administered with NAC (900 mg) twice daily or matching placebo for 3 months. Then, respiratory health status was evaluated using the St. George's Respiratory Questionnaire (SGQR), which was set as the primary end point.

**Results:**

A total of 143 COPD patients with chronic bronchitis were screened, and as a result, only 100 patients were enrolled in this study (50 participants were randomized to receive placebo, and others were randomized to receive NAC). After treatment, differences in SGQR scores between the placebo and NAC groups were not significant. Moreover, differences in secondary end points between the two groups after treatment were insignificant. *Discussion*. High-dose NAC has no marked clinical benefits for COPD patients with concurrent chronic bronchitis.

## 1. Introduction

Globally, chronic obstructive pulmonary disease (COPD) is a severe health challenge. Its prevalence in men and women is 9.2% and 6.2%, respectively [1]. For patients with late COPD, their job opportunities are severely limited, while their ability to engage in domestic, family, or social activities is impaired. Inhaled corticosteroids and inhaled long-acting bronchodilators are the two main treatment options for COPD patients. These drugs reduce disease progression; however, symptomatic or overall respiratory health improvements have not been reported. In most cases, these drugs did not improve the clinically important St. George's Respiratory Questionnaire (SGRQ) [2, 3].

If a COPD patient coughs for at least 3 months a year and for at least 2 years, he is considered to have chronic bronchitis, which is a common symptom in COPD patients [4]. Compared to patients with nonchronic bronchitis, when adjusted for age, gender, and airflow obstruction degree, chronic bronchitis patients have worse respiratory health and higher mortality rates. Therefore, it is important to develop new treatment methods for COPD patients [4].

The article "Efficacy and Safety of N-Acetylcysteine for Chronic Obstructive Pulmonary Disease and Chronic Bronchitis" was retracted in 2023. Reasons: signs of a paper mill; compromised peer review; unreliable results or conclusions.

Glutathione (GSH) is a tripeptide with anti-inflammatory and systemic antioxidant properties. Oral *N*-acetylcysteine (NAC) enhances GSH synthesis in the lungs, thereby improving clinical outcomes [5].

Globally, oral NAC is commonly used as a therapeutic option, and its efficacy has been verified in large clinical trials. It is usually administered at a dose of 300-1200 mg per day, and it may be effective in preventing COPD progression as well as in symptomatic improvement. However, the currently available clinical trials have not reported consistent findings [6–9]. NAC is also safe. Orally administered NAC (6000-8000 mg) to HIV infected people was not associated with any significant adverse effects [10]. Therefore, we hypothesized that a higher dose of NAC than the commonly used dose for COPD patients may improve clinical outcomes while remaining safe and tolerable.

## 2. Methods

### 2.1. Study Participants

This was a large randomized controlled trial involving COPD patients with sputum production and chronic cough. The inclusion criteria were as follows: (i) post-bronchodilator forced expiratory volume in 1 s (FEV_1_) less than 65% and ratio of FEV_1_ to forced vital capacity less than 0.70; (ii) between 20 and 75 years in age; (iii) a history of cigarette smoking more than 5 pack-years; (iv) within exacerbation of COPD during recent 3 months; and (v) Patients with chronic bronchitis. Chronic bronchitis was defined as sputum production “a few days a week” or “almost every day” and cough “a few days a week” or “almost every day” [11]. The exclusion criteria were as follows: (i) a primary diagnosis of asthma; (ii) cirrhosis with edema or ascites; (iii) received long-acting nitrate; and (iv) could not provide informed consent.

### 2.2. Randomization

Study participants were randomized at a ratio of 1 : 1 to a square of size 2 and administered with the active drug or placebo. “rnorm” function in R software was used generate the randomization list, which was only accessible to study pharmacists that accordingly assigned the therapies. Study participants were completely blinded to their assigned therapy.

### 2.3. Procedures

To prevent oxidation, tablets containing 900 mg NAC were sealed and packaged in an aluminum foil. The appearance, blistering, taste, and smell of the placebo and active drugs were comparable. For administration, patients were asked to dissolve the two tablets using fruit juice or just water twice a day. Treatment duration was 3 months. Patients were allowed to continue to use all conventional drugs, except guaiacol ether and other over-the-counter antitussive drugs.

The article "Efficacy and Safety of N-Acetylcysteine for Chronic Obstructive Pulmonary Disease and Chronic Bronchitis" was retracted in 2023. Reasons: signs of a paper mill; compromised peer review; unreliable results or conclusions.

### 2.4. End Points

The primary end point was the total SGRQ score, which is an effective method for measuring the health status of participants [11]. The SGRQ scores range from 0 to 100, of which 100 represents the worst respiratory health. Changes in three areas were assessed: SGRQ, Short Form-36 Health Survey (SF-36), and chronic bronchitis symptom assessment scale (CBSAS) as secondary end points [12, 13]. Pulmonary functions were assessed by the post-bronchodilator pulmonary function assay, and systemic oxidative stress was assessed by plasma 8-isoprostaglandin level, while systemic inflammation was assessed by evaluating serum C-reactive protein levels [14]. NAC-associated biochemical effects and oxidative stress were evaluated by assessing plasma changes of the mercaptan redox conjugate, cysteine/cystine, and GSH/GSH disulfide.

### 2.5. Statistical Analysis

The Shapiro-Wilk test was used to test whether data was normally distributed. For normally distributed data, chi-square tests and two-sided Student *t* test were used for baseline comparisons of treatment groups with regard to continuous and categorical variables, respectively. The highly skewed continuous and categorical variables were compared using the Wilcoxon signed-rank sum tests and Fisher's exact test, respectively. Statistical analyses were performed using SPSS, and *P* ≤ 0.05 was considered statistically significant.

## 3. Results

The participant selection process is shown in Figure 1. A total of 143 COPD patients with chronic bronchitis were screened, and as a result, only 100 patients were enrolled in this study (50 participants were randomized to receive placebo, while the others were randomized to receive NAC). As shown in Table 1, differences in baseline demographic characteristics between the two groups are not significant; however, SGQR scores in the NAC group (including symptoms, impacts, and total scores) are significantly lower, relative to the placebo group. After treatment, differences in the impacts became nonsignificant, while differences in the other two SGQR items remained significant (Figure 2). In terms of secondary end points, baseline SF-36 mental scores were balanced between the two groups, while after treatment, the SF-36 mental scores in the NAC group became significantly higher, relative to the placebo group (Figure 3).

The article "Efficacy and Safety of N-Acetylcysteine for Chronic Obstructive Pulmonary Disease and Chronic Bronchitis" was retracted in 2023. Reasons: signs of a paper mill; compromised peer review; unreliable results or conclusions.

## 4. Discussion

In this study, we found that high-dose NAC had no significant clinical benefits for COPD patients with chronic bronchitis.

The optimal method for evaluating the clinical symptoms associated with chronic bronchitis has not been determined. Therefore, we used changes in SGRQ total scores as the primary outcome. This is because, the SGRQ total score scheme is the most effective evaluation index for overall respiratory health of patients with COPD, and clinical significance differences of four units have been established.

Oral NAC is often described as a mucolytic agent because of its ability to cleave mucin disulfide bonds. *In vitro*, NAC, cysteine, and glutathione at equimolar concentrations of 50 mm markedly reduced mucus viscosity [5]. This effect was highly dose-dependent, and only a small effect was obvious after the 10th dilution. Glutathione concentrations in the alveolar epithelial lining fluid of smokers may be in the millimeter range; however, the real value may be much lower [15, 16]. Oral NAC can increase the concentration of GSH on the surface of alveoli and airways to reduce mucus viscosity; however, it has not been established whether this will bring important clinical benefits to patients with COPD and chronic bronchitis.

## Figures and Tables

**Figure 1:** Selection process of participants to the present study.

**Figure 2:** Differences in SGQR scores between the placebo and *N*-acetylcysteine groups after treatment. SGQR: St George's Respiratory Questionnaire.

**Figure 3:** Differences in CBSAS, SF-36-physical, and SF-36-mental scores between the placebo and *N*-acetylcysteine groups after treatment. SF-36: Short Form-36 Health Survey.

**Table 1:** Baseline characteristics of enrolled participants.

	Placebo (*N* = 50)	*N*-acetylcysteine (*N* = 23)	*P* value
Age, years (mean ± SD)	70 ± 5	71 ± 4	0.13
Sex, M/F	27/23	26/24	0.84
FEV_1_ (L), mean ± SD	1.15 ± 0.31	1.06 ± 0.23	0.11
SGQR (mean ± SD)			
Symptoms	70.5 ± 10.8	55.3 ± 10.7	<0.01
Activity	69.4 ± 13.4	69.9 ± 10.4	0.83
Impacts	43.8 ± 13.8	36.7 ± 11.9	<0.01
Total	55.7 ± 12.4	50.8 ± 9.5	0.03
CBSAS (mean ± SD)	2.2 ± 0.5	18.1 ± 4.2	<0.01
SF-36 (mean ± SD)			
Physical	37.1 ± 4.4	37.2 ± 3.9	0.91
Mental	49.6 ± 6.6	49.1 ± 7.4	0.71

M/F: male/female; FEV1: forced expiratory volume in the first second; SGQR: St. George's Respiratory Questionnaire; Short Form-36 Health Survey.

## Data Availability

No data were used to support this study.

## References

[1] Ntritsos G., Franek J., Belbasis L. (2018). Gender-specific estimates of COPD prevalence: a systematic review and meta-analysis. *International Journal of Chronic Obstructive Pulmonary Disease*.

The article "Efficacy and Safety of N-Acetylcysteine for Chronic Obstructive Pulmonary Disease and Chronic Bronchitis" was retracted in 2023. Reasons: signs of a paper mill; compromised peer review; unreliable results or conclusions.

[2] Calverley P. M., Anderson J. A., Celli B. (2007). Salmeterol and fluticasone propionate and survival in chronic obstructive pulmonary disease. *The New England Journal of Medicine*.

[3] Antoniu S. A. (2009). UPLIFT Study: the effects of long-term therapy with inhaled tiotropium in chronic obstructive pulmonary disease. Evaluation of: Tashkin DP, Celli B, Senn S et al.: a 4-year trial of tiotropium in chronic obstructive pulmonary disease. N Engl J Med (2008) 359(15):1543-1554. *Expert Opinion on Pharmacotherapy*.

[4] Kim V., Criner G. J. (2013). Chronic bronchitis and chronic obstructive pulmonary disease. *American Journal of Respiratory and Critical Care Medicine*.

[5] Sheffner A. L. (1963). The reduction *in vitro* in viscosity of mucoprotein solutions by a new mucolytic agent, N-acetyl-L-cysteine. *Annals of the New York academy of sciences*.

[6] Sutherland E. R., Crapo J. D., Bowler R. P. (2006). N-acetylcysteine and exacerbations of chronic obstructive pulmonary disease. *COPD*.

[7] Stey C., Steurer J., Bachmann S., Medici T. C., Tramèr M. R. (2000). The effect of oral N-acetylcysteine in chronic bronchitis: a quantitative systematic review. *The European Respiratory Journal*.

[8] Decramer M., Rutten-van Mölken M., Dekhuijzen P. N. (2005). Effects of N-acetylcysteine on outcomes in chronic obstructive pulmonary disease (bronchitis randomized on NAC cost-utility study, BRONCUS): a randomised placebo-controlled trial. *Lancet*.

[9] Zheng J. P., Wen F. Q., Bai C. X. (2014). Twice daily N-acetylcysteine 600 mg for exacerbations of chronic obstructive pulmonary disease (PANTHEON): a randomised, double-blind placebo-controlled trial. *The Lancet Respiratory Medicine*.

[10] De Rosa S. C., Zaretsky M. D., Dubs J. G. (2000). N-acetylcysteine replenishes glutathione in HIV infection. *European Journal of Clinical Investigation*.

[11] Jones P. W., Quirk F. H., Baveystock C. M. (1991). The St. George’s respiratory questionnaire. *Respiratory Medicine*.

[12] Au D. H., Blough D. K., Kirchdoerfer L., Weiss K. B., Udris E. M., Sullivan S. D. (2005). Development of a quantifiable symptom assessment tool for patients with chronic bronchitis: the chronic bronchitis symptoms assessment scale. *COPD: Journal of Chronic Obstructive Pulmonary Disease*.

[13] Tarlov A. R., Ware J. E., Greenfield S., Nelson E. C., Perrin E., Zubkoff M. (1989). The medical outcomes study. *JAMA*.

[14] Cracowski J. L., Durand T., Bessard G. (2002). Isoprostanes as a biomarker of lipid peroxidation in humans: physiology, pharmacology and clinical implications. *Trends in Pharmacological Sciences*.

[15] Cantin A. M., North S. L., Hubbard R. C., Crystal R. G. (1987). Normal alveolar epithelial lining fluid contains high levels of glutathione. *Journal of Applied Physiology*.

The article "Efficacy and Safety of N-Acetylcysteine for Chronic Obstructive Pulmonary Disease and Chronic Bronchitis" was retracted in 2023. Reasons: signs of a paper mill; compromised peer review; unreliable results or conclusions.

[16] Ward C., Thien F., Secombe J., Gollant S., Walters E. H. (2000). Bronchoalveolar lavage fluid urea as a measure of pulmonary permeability in healthy smokers. *The European Respiratory Journal*.

